The article "Inhibitory effect of Puerariae radix flavones on platelet-derived growth factor-BB-induced proliferation of vascular smooth muscle cells via PI3K and ERK pathways" was retracted in 2023. Reasons: plagiarized images; overlap with other authors' work; signs of a paper mill; concerns about the images.

# Inhibitory effect of *Puerariae radix* flavones on platelet-derived growth factor-BB-induced proliferation of vascular smooth muscle cells via PI3K and ERK pathways

**DOI:** 10.3892/etm.2014.2074

**Published:** 2014-11-17

**Authors:** HUI LI, KAIJUN LUO, JUAN HOU

**Affiliations:** Department of Immunology and Microbiology, Medical School of Jishou University, Jishou, Hunan 416000, P.R. China

**Keywords:** *Puerariae radix* flavones, vascular smooth muscle cell, platelet-derived growth factor-BB, proliferation

## Abstract

Abnormal proliferation of vascular smooth muscle cells (VSMCs) results in intimal thickening of the aorta, which may lead to arteriosclerosis. Therefore, VSMC antiproliferative agents may be efficient in the prevention and treatment of arteriosclerosis. *Puerariae radix* (PR) is the dried root of *Pueraria lobata* Ohwi or *Pueraria thomsonii* Benth. Flavones are the main components of PR and have been shown to have a protective effect on vascular disorders in traditional Chinese medicine treatments. However, the underlying molecular mechanism remains unclear. The aim of the present study was to explore the effect of PR flavone (PRF) on platelet-derived growth factor (PDGF)-BB-induced VSMC proliferation. PDGF-BB (25 ng/ml) and different doses of PRF (10, 50, 100 and 200 ng/ml) were used to treat VSMCs. The results revealed that PRF notably inhibited the PDGF-BB-induced VSMC proliferation and induced a cell cycle arrest at growth 1 phase of the cell cycle. In addition, cell cycle-associated proteins, including cyclin D1, proliferating cell nuclear antigen and cyclin-dependent kinase 4, were found to be downregulated. Furthermore, PRF inhibited the PDGF-BB-stimulated downregulation of VSMC markers, including α-smooth muscle actin, desmin and smoothelin. PDGF-BB upregulated the phosphorylation levels of phosphatidylinositide 3-kinase (PI3K) and extracellular signal-regulated kinase (ERK), which are associated with cell proliferation; however, these were decreased following PRF treatment. These observations indicated that PRF had a suppressive effect on PDGF-BB-induced VSMC proliferation by inhibiting PI3K and ERK pathways.

## Introduction

Abnormal proliferation of vascular smooth muscle cells (VSMCs) results in intimal thickening of the aorta, which may lead to arteriosclerosis and restenosis following percutaneous coronary intervention (PCI) or vein grafting (1,2). Therefore, VSMC antiproliferative agents may be effective in the prevention and treatment of vascular disorders.

*Puerariae radix* (PR), the dried root of *Pueraria lobata* Ohwi or *Pueraria thomsonii* Benth, has a sweet taste and is neutral in nature. PR can invigorate the spleen and stomach, and has been used in the prevention and treatment of vascular diseases in traditional Chinese medicine (3,4). Flavones are the main components of PR and have been previously shown to have a protective effect on arteriosclerosis (5). However, whether PR flavones (PRFs) have an inhibitory effect on VSMC proliferation remains unclear.

Platelet-derived growth factor (PDGF)-BB participates in vascular remodeling (6). The expression of PDGF-BB is know to be evidently increased following vascular injury, which further activates cell proliferation signaling by binding to PDGF receptor β (PDGFRβ) (7). Under physiological conditions, VSMCs remain in a quiescent state and express α-smooth muscle actin (α-SMA), desmin and smoothelin (8). However, in response to various stimuli, such as PDGF-BB, VSMCs may switch to a highly proliferative state, resulting in decreased expression levels of these markers (9). Furthermore, the cell cycle progression and expression levels of cell cycle-associated proteins have been found to be upregulated by PDGF-BB in VSMCs (10).

The aim of the present study was to determine whether PRF had an inhibitory effect on PDGF-BB-stimulated VSMC proliferation. In addition, the underlying molecular mechanism was investigated, including the phosphatidylinositide 3-kinase (PI3K) and extracellular signal-regulated kinase (ERK) pathways.

## Materials and methods

### Materials and agents

PRF was obtained from Anhui Joyfar Pharmaceutical Co., Ltd, (Bozhou, China), while Dulbecco’s modified Eagle’s medium (DMEM)/F12 and fetal bovine serum (FBS) were purchased from Life Technologies (Carlsbad, CA, USA). Dimethyl sulfoxide (DMSO), MTT and recombinant human PDGF-BB were purchased from Sigma-Aldrich (St. Louis, MO, USA). Mouse anti-cyclin D1, proliferating cell nuclear antigen (PCNA), cyclin-dependent kinase (CDK) 4, α-SMA, desmin, smoothelin, phospho-protein kinase B (Akt), total Akt, phospho-ERK, total ERK, glyceraldehyde 3-phosphate dehydrogenase (GAPDH) antibodies and rabbit anti-mouse secondary antibodies were obtained from Abcam (Cambridge, UK).

### Cell culture

VSMCs were isolated from the thoracic aortas of 10-week-old male Sprague-Dawley rats (obtained from the Animal Center of Jishou University, Jishou, China). The cells were cultured at 37°C in a humidified atmosphere (95% air, 5% CO_2_) using DMEM/F12 in 10% FBS. VSMCs at passage 5 were used in the study. The experiments of this study were approved by the Ethics Committee of Jishou University (Jishou, China) and were carried out according to the Guide for the Care and Use of Laboratory Animals (11).

### MTT assay

The VSMCs were cultured to 70% confluence and were serum-starved for 24 h in 96-well plates. The samples were divided into the following groups: control group (10 μl PBS), PDGF-BB group (25 ng/ml PDGF-BB) and four PDGF-BB + PRF groups with various PRF doses (25 ng/ml PDGF-BB and 10, 50, 100 or 200 ng/ml PRF). After culturing for 24 h, MTT (0.5 μg/ml) was added to the samples, followed by incubation for 2 h. Subsequently, the supernatant was removed using a pipette and 100 μl DMSO was added to dissolve the precipitation. The absorbance at 570 nm was determined using a Model 680 Microplate Absorbance reader (Bio-Rad Laboratories, Hercules, CA, USA).

### Cell cycle distribution analyses

The cell cycle distribution was determined using propidium iodide (PI) staining and flow cytometry (FACSCalibur; Beckman Coulter, Inc., Brea, CA, USA). The cells were fixed in 70% ethanol overnight at −20°C. Next, the cells were pelleted, washed in phosphate buffered saline (PBS) with 3% bovine serum albumin (BSA) and pelleted again. Subsequently, the cells were resuspended with PBS and incubated for 30 min at room temperature in PBS with 3% BSA, 40 μg/ml PI and 0.2 mg/ml RNase. The DNA content was determined by flow cytometric analysis.

### Western blot assay

Western blot assay was performed to determine the protein expression levels in each group. The cells were lysed in cold radioimmunoprecipitation assay buffer (Invitrogen Life Technologies, Carlsbad, CA, USA). A BCA Protein Assay kit (Thermo Fisher Scientific, Waltham, MA, USA) was used to determine the protein concentrations, according to the manufacturer’s instruction. Subsequently, the proteins were separated on a 10% sodium dodecyl sulphate-polyacrylamide gel and transferred to a polyvinylidene fluoride (PVDF) membrane. The PVDF membrane was blocked with 5% fat dry milk in PBS for 4 h. Subsequently, the PVDF membrane was incubated with specific primary antibodies (mouse anti-cyclin D1, mouse anti-PCNA, mouse anti-CDK4, mouse anti-smooth muscle-α-actin, mouse anti-smoothelin, mouse anti-desmin, mouse anti-phospho-Akt, mouse-anti-Akt, anti-phospho-ERK, mouse-anti-ERK, and mouse anti-glyceraldehyde 3-phosphate dehydrogenase antibodies; all from Abcam, Cambridge, UK) for 3 h. After washing three times with PBS (5 min each time), the PVDF membrane was incubated with a rabbit anti-mouse secondary antibody (Abcam). Next, after washing three times with PBS (5 min each time), an enhanced chemiluminescence western blotting kit (Thermo Fisher Scientific) was used to detect the immune complexes present on the PVDF membrane.

### Statistical analysis

The data are expressed as the mean ± standard deviation of three independent experiments and were analyzed using SPSS 17.0 statistical software (SPSS, Inc., Chicago, IL, USA). Statistical differences between the groups were determined using one-way analysis of variance. P<0.05 was considered to indicate a statistically significant difference.

## Results

### PRF inhibits PDGF-BB-induced VSMC proliferation

MTT assay was performed to investigate the effect of various PRF doses (10, 50, 100 and 200 ng/ml) on PDGF-BB-induced VSMC proliferation. The results indicated that the proliferation of VSMCs was notably increased following stimulation with 25 ng/ml PDGF-BB for 24 h, when compared with the PBS-treated control group. PRF doses between 10 and 200 ng/ml were found to inhibit the VSMC proliferation. The strongest inhibitory effect was achieved when using 100 ng/ml PRF; thus, this dose was selected for further experiments (Fig. 1).

### PRF suppresses the upregulation of cell cycle progression in PDGF-BB-treated VSMCs

The cell cycle is the series of events that take place in a cell leading to its division. Cells increase in size in the G1 phase and DNA replication occurs during S phase. Furthermore, the G1 checkpoint control mechanism ensures that everything is ready for DNA synthesis and thus controls cell cycle progression. In the current study, cell cycle progression was investigated in each group. The results revealed that PDGF-BB was found to promote cell cycle progression in VSMCs when compared to the control group. However, cells at growth 1 (G_1_) phase were found to be significantly upregulated in PDGF-BB + PRF-treated VSMCs compared with PDGF-BB-treated VSMCs, indicating that PRF induced a cell cycle arrest at G_1_ phase in PDGF-BB-stimulated VSMCs (Fig. 2A). In addition, changes in G_1_ phase arrest-associated proteins were investigated in each group. Cyclin D1, PCNA and CDK4 are cell cycle-associated proteins, participating in the regulation of the cell cycle between phases G_1_ and S. The expression levels of these proteins have been shown to be upregulated by PDGF-BB in VSMCs (10,12). Administration of PRF resulted in cell cycle arrest in PDGF-BB-treated VSMCs; thus, PRF may be involved in the expression level regulation of cyclins and CDKs in VSMCs. The western blot assay results indicated that the expression levels of cyclin D1, PCNA and CDK4 in PDGF-BB-treated VSMCs were significantly upregulated when compared with the control group. However, treatment with PRF notably inhibited the upregulation of cyclin D1, PCNA and CDK4 induced by PDGF-BB in VSMCs (Fig. 2B).

### PRF suppresses the PDGF-BB-induced proliferative phenotype switch of VSMCs

VSMCs have been shown to switch from a differentiated to a proliferative phenotype upon PDGF-BB stimulation, resulting in the downregulation of the VSMC differentiation markers, α-SMA, smoothelin and desmin (9). PRF was found to inhibit the PDGF-BB-stimulated proliferation of VSMCs; therefore, the expression levels of the aforementioned markers in the VSMC differentiated phenotype were investigated for each group. As demonstrated in Fig. 3, PDGF-BB significantly inhibited the protein expression levels of α-SMA, smoothelin and desmin in VSMCs, indicating that VSMCs dedifferentiated to a proliferative phenotype. However, the expression levels of these markers were found to be higher in PDGF-BB + PRF-treated VSMCs compared with PDGF-BB-treated VSMCs, indicating that PRF inhibited the PDGF-BB-induced proliferative phenotype switch in VSMCs.

### PRF inhibits the PDGF-BB-induced activation of PI3K and ERK pathways in VSMCs

PI3K and ERK pathways have been shown to play a crucial role in the regulation of cell proliferation (13). PDGF-BB may activate these two pathways in VSMCs (14). The results of the present study indicated that PRF inhibited the PDGF-BB-induced VSMC proliferation; therefore, PRF may have an effect on the activity of PI3K and ERK pathways. In order to verify this hypothesis, the activity of PI3K and ERK signaling pathways was investigated in PDGF-BB-treated VSMCs with or without administration of PRF. As shown in Fig. 4, the phosphorylation levels of Akt and ERK in PDGF-BB-treated VSMCs were significantly higher compared with the control group, indicating that these two signaling pathways were activated. However, the phosphorylation levels were notably decreased upon treatment with PRF. Therefore, the results of this study indicated that PRF suppressed the PDGF-BB-induced activation of PI3K and ERK pathways.

## Discussion

Vascular injury results in increased production of inflammatory factors and cytokines, such as PDGF-BB that has been demonstrated to play a promoting role in VSMC proliferation. In the present study, PDGF-BB was shown to significantly stimulate VSMC proliferation. Abnormal upregulation of VSMC proliferation induces neointima formation, which is closely associated with arteriosclerosis and restenosis following PCI or vein grafting. Inhibition of PDGF-BB-induced VSMC proliferation is crucial for the prevention of these vascular disorders (15). PR is the dried root of *Pueraria lobata* Ohwi or *Pueraria thomsonii* Benth, which has been used for the prevention and treatment of cardiovascular disease in traditional Chinese medicine (16). Previous studies have demonstrated that flavones are the main components of PR. PRF participates in coronary circulation, cardiac hemodynamics and myocardial metabolism (17). Furthermore, PR has been shown to have a protective effect on arteriosclerosis. Wu *et al* demonstrated that PRF significantly attenuated the development of advanced atherosclerotic plaques in a dose-dependent manner (5). In addition, the authors hypothesized that the underlying molecular mechanisms may be associated with decreased expression of caspase-3, as well as reduced apoptosis of macrophages in atherosclerotic plaques (5). Furthermore, Cai *et al* suggested that PRF may lower blood pressure and inhibit cerebral vascular resistance through the renin-angiotensin-system (18). However, the effect of PRF on PDGF-BB-induced VSMC proliferation, as well as the underlying molecular mechanism, have not been previously studied. To the best of our knowledge, the present study identified for the first time that PRF may effectively attenuate PDGF-BB-stimulated VSMC proliferation by inducing a cell cycle arrest at G_1_ phase and inhibiting the activation of PI3K and ERK pathways.

In the current study, PRF treatment was found to inhibit PDGF-BB-stimulated VSMC proliferation for the first time. VSMC proliferation is known to be closely regulated by cell cycle progression, where G_1_/S transition is a major control point in the initiation and completion of DNA replication (19,20). Therefore, the cell cycle progression was investigated in each group, and PRF was found to induce a cell cycle arrest at G_1_ phase in PDGF-BB-treated VSMCs. G_1_/S progression has been shown to be strongly mediated by the activity of the cyclin D1/CDK4 complex (21,22). Therefore, the expression levels of cell cycle-associated proteins were also investigated. PDGF-BB was found to significantly increase the expression levels of cyclin D1 and CDK4 in VSMCs, whereas administration of PRF had the opposite effect. In addition, the expression level of PCNA was found to be inhibited by PRF in PDGF-BB-treated VSMCs. PCNA plays an essential role in the regulation of DNA replication and cell proliferation. Three PCNA molecules can form a molecular sliding clamp around the DNA double helix, providing a platform for the dynamic recruitment and coordinated regulation of various proteins (23). Based on these observations, the inhibition of cyclin D1, PCNA and CDK4 expression levels may be closely associated with the inhibitory effect of PRF on PDGF-BB-stimulated VSMC proliferation.

In response to stimuli, such as PDGF-BB, VSMCs can dedifferentiate into a proliferative phenotype. Therefore, the effect of PRF on the PDGF-BB-stimulated VSMC phenotype switch was investigated. The results revealed that PDGF-BB notably inhibited the protein expression levels of three VSMC makers (α-SMA, desmin and smoothelin), indicating that VSMCs dedifferentiated into a proliferative phenotype. However, PRF treatment restored the marker expression levels in VSMCs. Therefore, the results indicate that PRF inhibited the PDGF-BB-induced VSMC proliferation by maintaining the differentiated phenotype of VSMCs.

Previous studies have demonstrated that PI3K and ERK pathways play a key role in the regulation of cell proliferation (13,24,25). Furthermore, the expression levels of cyclin D1, PCNA and CDK4 are regulated by these two signaling pathways (12,26,27). PI3K and ERK pathways are involved in the regulation of vascular remodeling, as well as VSMC proliferation. Fan *et al* showed that the PI3K/Akt signaling pathway plays a vital role in the modulation of cytoskeleton rearrangement and phenotype switching of pulmonary arterial smooth muscle cells (28). In addition, Yu *et al* hypothesized that ERK pathway may be involved in the pathogenesis of abnormal proliferation in rat pulmonary artery smooth muscle cells, as well as the rat pulmonary vascular remodeling induced by cigarette smoke exposure (29). Therefore, in the present study, the activity of PI3K and ERK pathways was determined in each group. The results revealed that PRF administration inhibited the upregulated activities of PI3K and ERK pathways in VSMCs treated with PDGF-BB. Therefore, the suppressive effect of PRF on the PDGF-BB-induced VSMC proliferation may be through inhibition of the PI3K and ERK pathway activation.

In conclusion, PRF was found to suppress PDGF-BB-induced VSMC proliferation by inducing a cell cycle arrest at G_1_ phase, inhibiting phenotype switching and suppressing the activation of PI3K and ERK pathways. Therefore, PRF may be a promising agent in the prevention and treatment of arteriosclerosis and restenosis following PCI or vein grafting.

## Figures and Tables

**Figure 1:** MTT assay showing the effect of PDGF-BB (25 ng/ml) and various doses of PRF (10, 50, 100 and 200 ng/ml) on cellular proliferation in vascular smooth muscle cells. ^**^P<0.01 compared with the two ends of the line. PDGF-BB, platelet-derived growth factor; PRF, *Puerariae radix* flavone.

**Figure 2:** (A) Cell cycle distribution in each group, determined using propidium iodide staining and flow cytometry. (B) Protein expression levels of cyclin D1, PCNA and CDK4, determined using western blot assay. GAPDH was used as the internal control. ^**^P<0.01 compared with the two ends of the line. Control, untreated VSMCs; PDGF-BB, VSMCs treated with 25 ng/ml PDGF-BB for 48 h; PDGF-BB + PRF, VSMCs treated with 25 ng/ml PDGF-BB and 100 ng/ml PRF for 48 h; VSMC, vascular smooth muscle cell; PDGF-BB, platelet-derived growth factor; PRF, *Puerariae radix* flavone; PCNA, proliferating cell nuclear antigen; CDK, cyclin-dependent kinase.

**Figure 3:** Protein expression levels of α-SMA, smoothelin, and desmin determined using western blot assay. GAPDH was used as the internal control. ^**^P<0.01 compared with the two ends of the line. Control, untreated VSMCs; PDGF-BB, VSMCs treated with 25 ng/ml PDGF-BB for 48 h; PDGF-BB + PRF, VSMCs treated with 25 ng/ml PDGF-BB and 100 ng/ml PRF for 48 h; VSMC, vascular smooth muscle cell; PDGF-BB, platelet-derived growth factor; PRF, *Puerariae radix* flavone; α-SMA, α-smooth muscle actin.

**Figure 4:** Protein expression levels of p-Akt, t-Akt, p-ERK and t-ERK determined by western blot assay. GAPDH was used as the internal control. In the graph, Akt refers to the p-Akt/t-Akt/GAPDH, and ERK refers to the p-ERK/t-ERK/GAPDH combined results, respectively. ^**^P<0.01 compared with the two ends of the line. Control, untreated VSMCs; PDGF-BB, VSMCs treated with 25 ng/ml PDGF-BB for 48 h; PDGF-BB + PRF, VSMCs treated with 25 ng/ml PDGF-BB and 100 ng/ml PRF for 48 h; VSMC, vascular smooth muscle cell; PDGF-BB, platelet-derived growth factor; PRF, *Puerariae radix* flavone; Akt, protein kinase B; EPK, extracellular signal-regulated kinase; p, phospho; t, total.
